# A Meta-Analysis of How Nonalcoholic Fatty Liver Disease Affect Antiviral Treatment of Patients with e Antigen-Positive Chronic Hepatitis B

This article has been retracted.

**DOI:** 10.1155/2022/4774195

**Published:** 2022-10-03

**Authors:** Yandong Chen, Qiang Liu, Jing Han, Siyu Gao, Qian Xiao, Xiaoli Huang, Lu Lu, xiaolin Zhou

**Affiliations:** Yichang Central People's Hospital, The First College of Clinical Medical Science, China Three Gorges University, Yichang, Hubei, China

## Abstract

**Background:**

Nonalcoholic fatty liver disease (NAFLD) and chronic hepatitis B (CHB) are both the most common underlying diseases leading to cirrhosis and hepatocellular carcinoma, and NAFLD and HBV infection are the first and second leading causes of chronic liver disease in China. However, there are still a lot of controversies about whether the combined presence of CHB and NAFLD will affect the course or outcome of liver disease together with HBV, and how the two affect each other.

**Objective:**

To investigate the effect of nonalcoholic fatty liver disease (NAFLD) on antiviral therapy in patients with chronic hepatitis B (CHB).

**Methods:**

Computer searches of databases such as PubMed, CNKI, VIP.com, and Wanfang Data Knowledge Service Platform were used. The time frame was from the creation of the database to June 2022. The search subject terms were hepatitis B, CHB, or NAFLD. The observation group consisted of patients with e antigen-positive CHB with NAFLD, and the control group consisted of patients with e-antigen + CHB. Extracts including title, name, date of publication, number of samples, antiviral drugs, and outcome indicators were used for Meta-analysis. Funnel plots were drawn to analyze literature bias.

**Results:**

Seven papers including 1348 patients with HBeAg + CHB (observation group: *n* = 547, control group: *n* = 801) were finally included.

**Results:**

Seven papers including 1348 patients with HBeAg + CHB (observation group: *n* = 547, control group: *n* = 801) were finally included. *Results*. Meta-analysis showed that CHB patients with NAFLD had lower efficacy than CHB patients after 48 weeks of antiviral treatment with nucleotide analogs, as measured by three outcome indicators HBV DNA conversion rate, ALT-normalization, and HBeAg conversion rate.

**Conclusion:**

NAFLD reduces the effect of antiviral therapy in CHB patients, and the clinicopathological features of patients with NAFLD combined with chronic hepatitis B are different from those of patients with chronic hepatitis B alone, so early diagnosis by liver histological examination should be actively performed and reasonable antiviral therapy should be administered.

## 1. Introduction

NAFLD is one of the chronic liver diseases that has become one of the major chronic liver diseases in China and the most common chronic liver disease in the world, which is associated with insulin resistance and also with genetic susceptibility to liver damage when metabolic stress is produced, characterized by hepatic steatosis, and its disease spectrum includes from simple steatosis, nonalcoholic steatohepatitis, cirrhosis and cryptogenic cirrhosis [1, 2]. When NAFLD progresses to NASH, the risk of death increases, as it can develop cirrhosis and even liver cancer. In China, the main cause of cirrhosis is chronic hepatitis B, and more than 50 million people die each year from hepatitis B and from its complications, mainly liver failure and or hepatocellular carcinoma [3, 4]. Chronic hepatitis B is the most common chronic liver disease in China, but over the 30 years of reform and opening up, the standard of living has been improving, so people's lifestyles are changing, and NAFLD has become the leading cause of chronic liver disease in China, and the number of patients with the combination of both has increased [5].

In Western countries, the prevalence of NAFLD in the general population is about 30%, and the prevalence is even higher in obesity. The prevalence of NAFLD has been reported to affect 80–100 million people in the United States, of which 10–22% may develop NASH [6, 7]. The prevalence of NAFLD is increasing especially in Asian countries such as China and Japan, and the age is getting younger. One study showed that the rate of CHB combined with NAFLD was 18% to 62% in Europe and the Middle East and 14% to 17% in the Asia-Pacific region[8]. A study of 1309 patients with CHB in rural China with follow-up showed that the prevalence of combined NAFLD in patients with CHB increased from 6.40% in the year 2008 to 21.54% in the year 2012 in a 4-year period from 2008 to 2012, showing an increasing trend year by year [9].

Antiviral therapy is crucial for disease progression in CHB patients, and in recent years, antiviral therapies have been widely used in the clinic, and this modality has achieved notable success in the treatment of chronic hepatitis B. Data [10] showed that hepatic degeneration, hepatocellular neoplasm, positive hepatocellular neoplasm, and serum hepatitis B virus DNA levels were significantly reduced in steatosis patients, suggesting a protective effect of steatosis against lipofuscinosis. The study [11] demonstrated that NAFLD inhibits HBV without affecting host lipid homeostasis. However, the study [12] reported that antiviral therapy was ineffective in CHB patients with high CAP (controlled attenuation parameter). Therefore, there is controversy about how NAFLD affects CHB.

Based on this, in order to investigate the clinical effect of a simple antiviral method for chronic hepatitis B, computerized searches of PubMed, CNKI, VIP.com, and Wanfang Data Knowledge Service Platform databases were used in conjunction with the actual situation. The time range was from the establishment of the database to June 6, 2022. The keywords were Chinese search subject headings: hepatitis B, CHB, or NAFLD. English subject headings: Chinese and Red Cross, NAFLD. The observation group consisted of patients with *e* antigen-positive CHB, and the control group consisted of patients with *e*-antigen + CHB. Extracts including title, name, publication date, sample number, antiviral drug, and outcome index were used for Meta-analysis. Funnel plots were drawn to analyze literature bias. It is reported below.

## 2. Materials and Methods

### 2.1. Literature Search

Databases such as PubMed, CNKI, VIP.com, and Wanfang Data Knowledge Service Platform were searched using computers. The time range was from database creation to June 6, 2022. The keywords were Chinese search subject headings: hepatitis B, CHB, or NAFLD. English subject headings: Chinese and Red Cross, NAFLD. The observation group consisted of patients with *e* antigen-positive CHB, and the control group consisted of patients with *e* antigen + CHB. Extracts including title, name, publication date, sample number, antiviral drug, and outcome index were used for Meta-analysis. Funnel plots were drawn to analyze literature bias.

### 2.2. Inclusion Criteria

Inclusion criteria were as follows: the observation group of the research objects is the CHB patients with NAFLD who are positive for e antigen. The control group was CHB patients with positive e-antigen; study type: cohort study or case-control study; outcome indicators: serum HBV DNA level decreased to below 3 lg IU/mL, ALT normalized, and HBeAg negative conversion.

### 2.3. Exclusion Criteria

Exclusion criteria were as follows: (1) full text not available; (2) incomplete data; (3) duplication in the literature; (4) conclusion that the indicators do not match.

### 2.4. Data Extraction

The extracted content includes the title, first author, publication year, subject numbers, antiviral drugs, and outcome indicators.

### 2.5. Statistical Analysis

Statistical software 5.3 was used and *P* < 0.05 was considered statistically significant. RR and its 95% CI were chosen as statistical data. Heterogeneity between the literature was tested by the P test and the I^2^ test. *P* < 0.05 and I^2^ < 50% indicated that the literature was homogeneous (no heterogeneity) and a fixed-effects model was used, otherwise a random-effects model was used.

## 3. Results

### 3.1. Publication Screening

A computer search of databases such as PubMed, CNKI, VIP.com, and Wanfang Data Knowledge Service Platform. The time range was from the establishment of the database to June 6, 2022. Keywords: hepatitis B, nonalcoholic hepatitis. A total of 7 articles were included, including 1348 HBeAg + CHB patients, 547 observation cases, and 801 controls. The screening flow chart is shown in Figure 1, the characteristics of the literature are listed (Table 1), and the evaluation quality is shown in Table 2.

### 3.2. HBV DNA Negative Conversion

As shown in Figure 2, all 7 publications had the data of HBV- conversion after 48-week of antivirus. Statistical analysis found that 7 publications had a very small heterogeneity, so a fixed-effect model was adopted. Data indicated that HBV- conversion in CHB patients with NAFLD after 48-week of antiviral treatment was significantly decreased than in CHB patients.

### 3.3. ALT Normalization

As shown in Figure 3, all 7 studies provided data on the normalization of ALT after 48 weeks of antiviral treatment. Statistical analysis found a small heterogeneity among publications, so a fixed-effect model was adopted. Data demonstrated that the ALT-normalization rate in CHB patients with NAFLD after 48-week of antiviral treatment was lower than that in CHB patients.

### 3.4. HBeAg Negative Conversion

As shown in Figure 4, all 7 studies provided the data of HBeAg negative conversion after 48 weeks of antiviral treatment. Statistical analysis found that 7 publications had a very small heterogeneity, so a fixed-effect model was adopted. Data indicated that the HBeAg rate of CHB patients with NAFLD after 48-week of antiviral treatment was lower than CHB patients.

### 3.5. Literature Bias Analysis

A funnel plot analysis was performed on the rate of HBV conversion in the included literature (Figure 5).

## 4. Discussion

Chronic hepatitis B refers to a chronic disease characterized by the degree of hepatocellular damage after infection with hepatitis B [3]. Chronic disease is characterized by the degree of hepatocellular damage as the main pathological change after the infection [15, 16]. The disease is characterized by the degree of damage to liver cells. When the regulation of the body's immune system is disturbed, the patient's liver cells are damaged, resulting in liver damage. In the case of NAFLD, the liver cells are damaged, resulting in abnormal liver function and liver fibrosis. NAFLD is a liver disease caused by genetic predisposition and insulin resistance. NAFLD is a disease of liver parenchyma caused by excessive fat content in the liver cells due to genetic predisposition and insulin resistance. To some extent chronic hepatitis B and NAFLD are two separate diseases [17, 18], they often appear in a combined form and have a more pronounced effect on each other, leading to liver fibrosis. The two diseases are often combined and have a significant impact on each other, leading to liver fibrosis, which can accelerate cirrhosis if the patient does not receive the relevant treatment in the first place. If the patient does not receive the relevant treatment in the first place, the transformation process of cirrhosis will be accelerated, which is undoubtedly a great difficulty for clinical treatment. This is undoubtedly a great difficulty for clinical treatment.

The results of this study showed that the patients' AST, TG, TC, and ALT improved more significantly when they were treated with hepatoprotective therapy and the observation group was treated with antiviral therapy alone. Although the basic hepatoprotective therapy could improve liver function, fibrosis level, and ballooning changes to some extent, the effect was more significant with the addition of the antiviral method, and the patients were able to achieve 89% and 100% of the liver function level and HBV DNA conversion rate after the treatment [19].

It has been noted in the literature that there is also variability in the effectiveness of the use of antiviral treatment in patients with different NAFLD scores. Here among them the biochemical parameters of the 7 and 8 subgroups improved significantly compared to the pretreatment period, while the effect of antiviral therapy was more significant in patients with scores of 5–6. This fundamentally confirms that there is a correlation between the severity of fatty liver disease and the effectiveness of antiviral treatment for hepatitis B. The NAFLD score has a significant impact on the effectiveness of antiviral treatment for chronic hepatitis B disease. It is recommended that for this group of patients, intensive NAFLD treatment is used, which includes specific measures such as medications and exercise.

Treatment of CHB includes antiviral therapy with interferon and nucleoside analogs. Due to different mechanisms, we included only patients receiving antiviral therapy with nucleoside analogs. A total of 7 publications, including 1348 HBeAg + CHB patients with NOS score ≥ 7, were included and were of high quality. The meta-analysis finally concluded from the perspective of three outcome indicators, HBV-conversion, ALT-normalization, and HBeAg conversion, that CHB patients with NAFLD had lower efficacy than CHB patients after 48 weeks of antiviral therapy with nucleoside analogs. This is consistent with the results observed in most of the literature.

However, this meta-analysis has some drawbacks and limitations.

1. Antiviral treatment with nucleoside analogs is a long-term process. Due to the different follow-up time points of the included studies, this meta-analysis only examined the virological and biochemical responses after 48 weeks of antiviral therapy. However, there was a significant correlation between the duration of antiviral treatment and its response. Therefore, other experiments are needed to observe the efficacy at other time points.
2. Through a literature search, we retrieved 16 relevant studies, but because 9 of them did not specify the e-antigens of the included patients, no comprehensive analysis was performed. Only 6 papers were included for analysis, which is not a large enough sample size and may be potentially biased.

In patients with more severe fatty liver disease, the implementation of antiviral therapy can improve the overall liver function of the patient; thus, enabling the demonstration that the combination of antiviral therapy for those with poor hepatoprotective therapy alone can promote disease regression. For NAFLD scores of 5 to 6, patients with liver function ALT greater than 3NLN are recommended to be treated with simple antiviral therapy. This can reduce the liver load to some extent.

In conclusion, our study suggests that NAFLD inhibits antiviral therapy in patients with CHB. More experiments with larger samples are still needed to draw more accurate conclusions.

## 5. Conclusion

In conclusion, in patients with chronic hepatitis B combined with NAFLD, the use of hepatoprotective therapy along with antiviral therapy can improve the overall HBV DNA and HBsAg conversion rate, as well as liver function, improve NAFLD classification, better repair the degree of liver damage, and improve liver function, which is worth further promotion in clinical treatment. It is worth to further promote its use in clinical treatment.

## Figures and Tables

**Figure 1:** Literature screening process.

**Figure 2:** Data of HBV DNA negative conversion after 48-week antivirus.

**Figure 3:** Data of ALT normalization after 48-week antivirus.

**Figure 4:** Data of HBeAg negative conversion after 48-week antivirus.

**Figure 5:** Funnel plot analysis of the negative conversion rate of HBV DNA in the included literature.

**Table 1:** Literature's Basic characteristics.

First author	Issuing time (year)	Antiviral drugs	Total number of n	Observation group/control group	HBV DNA Yin turn (observation group/control group)	ALT return to normal (observation group/control group	HBeAg negative conversion (observation group/control group)
XI Jin [13]	2012	ETV	213	65/148	35/100	38/105	12/33

Li-Yao Zhu [14]	2016	ETV	125	61/64	38/48	40/52	13/15

Sun Jianmin [8]	2015	ETV	62	32/30	24/26	20/26	11/13

Wang Yanling [9]	2016	ADV	204	82/122	56/97	58/102	15/32

Wang Hao [10]	2019	ETV	273	123/150	113/141	100/135	24/44

Chen Xi [11]	2021	ETV	289	102/187	81/157	71/150	8/10

Wang Hao [12]	2018	TDF	182	82/100	75/94	65/90	14/29

*Note.* ETV: entecavir; TDF: tenofovir; ADV: adefovir dipivoxil.

**Table 2:** Literature quality NOS scale.

First author	Time of publication	Research object selection				Comparability between groups	Exposure factor measurement			Total score
		1	2	3	4		a	b	c	
XI Jin	2012	^*∗*^	^*∗*^	^*∗*^	^*∗*^	^*∗∗*^	^*∗*^	^*∗*^		8
Li-Yao Zhu	2016	^*∗*^	^*∗*^	^*∗*^	^*∗*^	^*∗*^	^*∗*^	^*∗*^		7
Sun Jianmin [8]	2015	^*∗*^	^*∗*^	^*∗*^	^*∗*^	^*∗∗*^	^*∗*^	^*∗*^		8
Wang Yanling [9]	2015	^*∗*^	^*∗*^	^*∗*^	^*∗*^	^*∗∗*^	^*∗*^	^*∗*^		8
Wang Hao [10]	2019	^*∗*^	^*∗*^	^*∗*^	^*∗*^	^*∗∗*^	^*∗*^	^*∗*^		8
Chen Xi [11]	2021	^*∗*^	^*∗*^	^*∗*^	^*∗*^	^*∗*^	^*∗*^	^*∗*^		7
Wang Hao [12]	2018	^*∗*^	^*∗*^	^*∗*^	^*∗*^	^*∗∗*^	^*∗*^	^*∗*^		8

*Note.* a determination of exposure factors; *b* use the same method to determine exposure factors of cases and control groups; *c* nonresponse rate; 1 Whether the determination of cases is appropriate; 2 Representation of cases; 3 Selection of control groups 4. Controls Sure.

## Data Availability

The data used to support the findings of this study are available from the corresponding author upon reasonable request.
